The article "Experimental Study on Interfacial Bond Behavior between CFRP Sheets and Steel Plates under Fatigue Loading" was published in 2019. Journal: Materials (Basel).

# Experimental Study on Interfacial Bond Behavior between CFRP Sheets and Steel Plates under Fatigue Loading

**DOI:** 10.3390/ma12030377

**Published:** 2019-01-25

**Authors:** Long Zhang, Shuangyin Cao, Xin Tao

**Affiliations:** 1 Key Laboratory of Concrete and Prestressed Concrete Structures of Ministry of Education, Southeast University, Nanjing 210096, China; 230129147@seu.edu.cn; 2 Nanjing Power Supply Company, Nanjing 210008, China; 230129148@seu.edu.cn

**Keywords:** carbon fiber-reinforced polymer, steel, interface, fatigue crack, fatigue life

## Abstract

Using carbon fiber reinforced polymer (CFRP) composites for enhancing the fatigue behavior of the steel structures will be an important application. As the most critical part, the fatigue behavior of the CFRP-to-steel bonded interface directly determines the strengthening effect of steel structures reinforced by CFRP. In this paper, a series of CFRP-to-steel double-shear specimens are performed in order to study the interfacial bond behavior between CFRP and steel under fatigue loading. Two parameters are considered: the upper bound value and the lower bound value of the fatigue loading. An analysis of test results indicates that the crack development rate increases with the increment of the stress ratio or stress level and the crack development process includes two phases: crack stable development phase and debonding failure phase. A calculation model is put forward to describe the relationship between the crack development rate and the stress level. Besides, it can be obtained from the test results that the fatigue lives of the specimens decrease with the increment of the stress level. The empirical formula of *S-N* curve based on the form of single logarithm formula is proposed and the fatigue limit under the experimental conditions in this paper is determined to be 0.343 by computational analysis.

## 1. Introduction

In current engineering, there are masses of defective steel structures that cannot meet the requirement of the design and operational caused by construction defects, environmental corrosion, and long-term cyclic loading. These defective steel structures urgently need to be strengthened and repaired. During the last few decades, fiber reinforced polymer (FRP) composites, and especially for carbon fiber reinforced polymer (CFRP) composites, have gained more and more attention in the strengthening engineering of structures for its high strength-to-weight, stiffness-to-weight ratios and corrosion resistance [1,2,3,4,5,6,7,8,9,10]. In the meanwhile, as the most critical part, the bond behavior of the bonded interfaces between CFRP and steel directly determines the reinforcement effects of a steel structure reinforced by CFRP [11]. Current studies about the bond behavior of CFRP-to-steel bonded interfaces under static loading have been carried out [12,13,14,15,16,17]. In particular, fatigue failure is one of the primary failure modes for steel structures under cyclic loading. Consequently, it is highly necessary to conduct thorough research on the fatigue performance of the bonded interfaces between CFRP and steel under cyclic loading. 

In comparison to concrete structures, the application of the use of CFRP to reinforce steel structures is still at an initial stage. In recent years, externally bonded CFRP sheets have proven to be significantly effective in improving fatigue performance and extending the fatigue life of steel elements [11,18,19,20,21]. However, there are few publications on the interfacial bond behavior between CFRP and steel subjected to fatigue loading. Liu et al. [22] investigated the effect of fatigue loading on the bond strength, bond slip and failure modes of CFRP bonded steel plate joints through a series of tests of CFRP double strapped bonded steel plate joints under fatigue loading. They found that when the upper bound value of the fatigue loading is less than 40% of the ultimate static strength there is no fatigue failure in the specimens. When the upper bound value of the fatigue loading is less than about 35% of the ultimate static strength, the influence on the bond strength is not significant (less than 10%). A reduction in bond slip stiffness was observed due to accumulated damage caused by the fatigue loading. The failure modes were not affected much by the fatigue loading except for those bonded with high modulus CFRP, where fiber fracture extended over more than one cross-section. Matta et al. [23] conducted a series of fatigue tests on steel/CFRP double strap adhesively-bonded specimens. The results showed that the fatigue resistance of the joints was at least comparable with that required for welded cover plates. The bond strength reduced to 83%–88% of that of unfatigued specimens and the stiffness was found to gradually reduce. Yang et al. [24] carried out 24 double-shear pull-out tests to study the fatigue behavior of the bonded joints. The test results indicated that the region of the joints around the loaded end presented degradation reflected on the bond-slip stiffness and on the increment of residual deformation. The interfacial stiffness of the adhesively bonded joints degraded with the number of cycles imposed on the specimens. Colombi et al. [25] carried out fatigue tests on CFRP-to-steel double strap bonded joints and found that the stiffness of the joints decreased with fatigue load due to the gradual debonding of the CFRP sheet. The initial fatigue crack was observed when the stiffness dropped to 98%, quicker debonding was associated with a stiffness reduction to 95%, and final failure occurred when the stiffness dropped to 90% of the initial value. Wu et al. [26] performed a series of fatigue tests on ultra high modulus (UHM) CFRP-to-steel double strap bonded joints and found that the bond strength decreased with the increment of the load ratio. Meanwhile, it was revealed from the microscope images of the fracture surface that the fatigue loading only introduced damage which was constrained within a very small zone close to the joint. This zone was named the “fatigue damage zone”, and 99% of the bond-line remained intact from the fatigue loading. 

Relevant studies on interfacial bond behavior between CFRP and steel structure under fatigue loading are very scarce and far from comprehensive. Meanwhile, the evolution law of interfacial fatigue crack is always analyzed based on the fracture mechanics, which is rather complicated and inconvenient to apply. In this paper, a series of CFRP-to-steel double-shear specimens were tested under fatigue loading by considering two key parameters—namely, the upper bound value and the lower bound value of the fatigue loading—and the fatigue performance of the adhesive interface between CFRP sheets and steel plates was analyzed. The experimental phenomena, CFRP strain distribution, interfacial crack propagation behavior, and fatigue life were discussed. On this basis, the relationship between the interfacial crack development rate and fatigue stress level, *S*-*N* curve empirical formula, as well as the Goodman–Smith Diagram were obtained in this paper.

## 2. Experimental Program

### 2.1. Materials

In this paper, the normal modulus CFRP sheets with a nominal thickness of 0.167 mm and the matched epoxy resin adhesives were supplied by NJMKT Corp (Nanjing, China). The type of this CFRP sheets is MKT-CFC300 with a matrix composed by an epoxy resin. According to the product date sheet, the nominal elastic modulus and tensile strength of the CFRP sheets were 240 GPa and 3529.1 MPa, respectively. The mixing ratio of the adhesive was 4:1 of epoxy resin to special filler by weight. The shear strength and nominal elastic modulus of the adhesive were 17.7 MPa and 2737.3 MPa, respectively. The steel plates, which had a thickness of 5 mm, were made of A283GRD steel (ASTM). The Young’s modulus and yield strength of the steel plates were 201 GPa and 263 MPa respectively. Material properties of CFRP sheets and epoxy resin adhesive are shown in Table 1.

### 2.2. Specimen Details

In order to make a thoroughly research on the fatigue performance of the adhesive interface between CFRP and steel, a total of 10 double-shear specimens were prepared in this study. The geometry and the dimensions of the specimens are illustrated in Figure 1. As show in Figure 1, two steel plates with a separation of 2 mm were connected by pasting CFRP sheets onto the both sides. The nominal width and the thickness of the CFRP sheets were 40 mm and 0.167 mm, respectively. In order to observe the whole process of the debonding failure, the specimens were designed, and consisted of two parts: a testing part with a bond length of 200 mm and a strengthened part with a bond length of 230 mm. The existence of the strengthened part ensured that the debonding failure occurred at the testing part firstly.

In the preparation of the specimens, the surface of the steel plate was first ground to create a clean, rough, and chemically active surface by using an electric angle grinder. Next, the bonded surfaces of both CFRP sheets and steel plates were further cleaned by using a large amount of acetone to wash off the fine abrasive dust. After bonding the CFRP sheets, the specimens were mechanically rolled to remove air bubbles and excess epoxy to create a uniform, thin layer of adhesive in order to offer ideal conditions to obtain a strong mechanical bond. All the specimens were cured in an indoor environment for seven days before testing [14].

The basic conditions of the specimens are shown through using combinations of the numbers and letters. In the acronym “*S (F)-L-W-R*_max_*-R*_min_”, “*S*“ and “*F*” stand for the static loading method and fatigue loading method, respectively. Additionally, “*L*” and “*W*” represent the bond length (*l*_c_) and the bond width (*b*_c_) (in mm) of the CFRP sheet in the testing part, respectively, while “*R*_max_” and “*R*_min_” represent the ratio of the upper bound value and of the lower bound value of the fatigue loading to the debonding load (*P*_k_) of each static specimen, respectively. Two groups of specimens, groups A and B, were designed by considering the influence of *R*_max_ and *R*_min_ on the fatigue performance of the adhesive interface between CFRP and steel, respectively. Details and test results of each specimen are detailed in Table 2.

### 2.3. Test Procedure

Both quasi-static loading and cyclic loading tests were performed by using an MTS (Material Testing System) fatigue machine (MTS Systems Corp, Eden Prairie, MN, USA) with a maximum measurement range of 10 tons in the Nanjing University of Technology (NUT). The quasi-static loading tests were conducted at a rate of 0.2 mm/min until failure in order to determine the debonding load of the CFRP sheets (*P*_k_) of each specimen. A constant-amplitude sinusoidal loading was applied to each cyclic specimen at a frequency of 10 Hz in the tension–tension fatigue test. The ratios of the upper bound value *R*_max_ and the lower bound value *R*_min_ of each cyclic specimen are listed in Table 2. Static preloading from zero loading to the upper bound value *P*_max_ was conducted at a rate of 0.2 mm/min on each cyclic specimen before cyclic loading to reduce the test error.

In order to obtain the evolution of the strain on the CFRP sheets both in the static and cyclic loading tests, the strain gauges were placed continuously on the surface of the CFRP sheets with a spacing of 15 mm along the centerline in the testing part. A DH3817 multichannel dynamic strain recorder (Beijing Hongchangxin Technology Co., Ltd, Beijing, China) was used for the strain collection. The test loading device and strain acquisition system are shown in Figure 2.

## 3. Experimental Results and Discussion

### 3.1. Testing Phenomenon 

For the specimens under static loading, the strain on the CFRP sheets increased steadily with the increment of load, and the specimens showed a good elastic property in the initial stage. The interfacial debonding initiated at the mid-span in the testing part of the specimen and was accompanied by a faint peeling sound when the load increased to about 85% of the ultimate load. Thereafter, the debonding proceeded toward the loaded end of the specimen and both the strain of the CFRP and the load remained about the same. The failure occurred suddenly with a loud noise when the debonding extended to the end of the CFRP sheets near the loaded end. The typical failure mode of the static specimens mainly occurred in the adhesive layer, as shown in Figure 3a. The test results in this paper are similar to those observed in a previous static test [27].

For the specimens subjected to cyclic loading, there were no obvious phenomena in the initial cyclic loading stage. Subsequently, the interfacial bond property between CFRP sheets and steel plates degraded with an increasing number of cycles and was accompanied by a faint peeling sound. The initial fatigue crack occurred at the mid-span in the testing part of the specimen when the number of cycles increased to a certain number, as shown in Figure 4. After that, the fatigue crack gradually propagated with an increase in the number of loading cycles from the mid-span to the loaded end of the specimen. Eventually, after a loud noise, failure occurred suddenly when the fatigue crack expanded to the end of the CFRP sheets near the loaded end. As shown in Figure 3b, cohesive failure within the adhesive layer was observed in cyclic tests. The specimens exhibited a gradual debonding process and showed good ductility. In previous study, the cohesive failure was regarded as the desired failure mode for the bonding interface between CFRP and steel [6], since the strength of the adhesive was efficiently used.

### 3.2. Strain Distribution of CFRP Sheets Along Bonding Length

The typical strain distribution of the CFRP sheets along the bonding length subjected to cyclic loading is shown in Figure 5. Each curve in Figure 5 represents the strain distribution of the CFRP sheets along the bonding length under the upper bound value *P*_max_ when the number of cycles increases to a certain number. 

As shown in Figure 5, a large strain gradient only occurs near the mid-span in the testing part of the specimens before interfacial debonding, which indicates that the deformation is mainly concentrated near the mid-span. A general trend is observed that the strain of the CFRP sheets always decreases rapidly with the increment of the distance away from the mid-span, and the trend is consistent at different number of cycles. The interfacial bond property between CFRP sheets and steel plate degrades with increasing number of cycles, which causes the capacity of the interfacial shearing stress transfer to get weakened, and the strain of the CFRP sheets attenuates slowly near the mid-span of the specimen. After interfacial debonding, the interfacial shearing stress can only be transferred by the friction of the interface in the debonding zone which enlarges gradually from the mid-span to the loaded end with increasing number of cycles, until eventually failure occurs. It is also observed that the maximum strain of the CFRP sheets at different number of cycles remains relatively constant in this process.

## 4. Evolution Law of Interfacial Fatigue Crack

### 4.1. Crack Propagation

Based on the analyses, the interfacial fatigue crack propagated gradually with increasing number of cycles. Obviously, the strain of the CFRP sheets at the point that the interfacial crack extended to should be equal to the strain in the debonding zone under the ideal condition. Meanwhile, the interfacial fatigue crack length “*a*” should be equal to the distance from the mid-span to the point that the crack extended to. However, due to the existence of mechanical interaction, local inhomogeneity of CFRP sheets, and the interfacial friction, the strain of CFRP sheets in the debonding zone was difficult to keep equal in the actual experiment. Therefore, in this paper, it could be regarded that the interfacial crack had extended to the point “z” if the strain of the CFRP sheets at the point “z” increased to be close to the strain in the debonding zone and changed very little with the increasing number of cycles. Based on this, the relationship of interfacial crack length “*a*” and number of fatigue cycles “*N*” could be obtained, as shown in Figure 6. 

It can be seen from Figure 6 that the curves of the specimens approximately present two stages. The first stage is a period of stable crack development. The crack length increases slowly with the increase of fatigue cycles in this stage. From the test results, the first stage can nearly reach to 95% of the fatigue life. For the specimens for which the upper bound value is less than 0.7*P*_k_ (F200-40-0.35-0.1, F200-40-0.4-0.1, F200-40-0.5-0.1, and F200-40-0.6-0.1), the crack length increases almost linearly with the increase of fatigue cycles in the first stage. However, for the specimens with an upper bound value of 0.7 *P*_k_ (F200-40-0.7-0.1, F200-40-0.7-0.2 and F200-40-0.7-0.3), the initial crack length of the CFRP sheets increases relatively faster with the increase of fatigue cycles. This is due to the fact that the initial crack development is less affected by the stress concentration at the mid-span when the upper bound value is less than 0.7*P*_k_. After the upper bound value nearly reaches to 0.7*P*_k_, the impact of the stress concentration on the initial crack development become larger, which leads to the phenomenon that the initial crack length increases relatively faster. After that, the crack development rate slows down and tends towards stability.

The second stage is the debonding failure period. In this stage, with the crack development, the remaining bond length of the CFRP sheet is less than the effective bonding length, and then debonding failure occurs suddenly because there is not sufficient resistance debonding bearing capacity. 

### 4.2. Crack Development Rate

The crack development rate of the interface between CFRP sheet and steel plate (*v*_cr_) can be calculated by the following equation:

*v*_cr_ = d*a*/d*N* (1)

where *a* and *N* indicate the crack length of the interface and the fatigue cycles, respectively. Based on the analysis result of the crack propagation in front, the first stage of the crack propagation can reach nearly 95% of the failure life. Meanwhile, for the specimens with an upper bound value of 0.7 *P*_k_ (F200-40-0.7-0.1, F200-40-0.7-0.2, and F200-40-0.7-0.3), the impact of initial stress concentration on the crack propagation only occupies less than 10% of the failure life. Therefore, the impact of initial stress concentration and the crack development rate of the second stage will not be discussed in this paper. For the first stage, the crack development rate is equal to the reciprocal of the curve in Figure 6. The crack development rate of each specimen was calculated as shown in Table 3.

It can be seen from Table 3 that the crack development rate (*v*_cr_) has a close relation with the upper bound value and the lower bound value of the fatigue loading. In this paper, stress ratio (*R*) and stress level (*S*) of fatigue loading will be discussed as the main parameters impacting on the crack development rate (*v*_cr_).

The stress ratio *R* can be expressed by:

(2) $$R=\frac{P_{\max}}{P_{\min}}$$

where *P*_max_ and *P*_min_ represent the upper bound value and the lower bound value of the fatigue loading, respectively. 

The stress level *S* can be expressed by:

(3) $$S=\frac{\Delta S}{1-S_{a}}$$

where *ΔS* represents the standardized stress amplitude of the CFRP sheet and can be expressed by:

(4) $$\Delta S=\frac{\sigma_{\max}-\sigma_{\min}}{\sigma_{k}}=\frac{P_{\max}-P_{\min}}{P_{k}}$$

*S*_a_ represents the standardized mean stress amplitude of the CFRP sheet and can be expressed by:

(5) $$S_{a}=\frac{\sigma_{\max}+\sigma_{\min}}{2\sigma_{k}}=\frac{P_{\max}+P_{\min}}{2P_{k}}$$

where *σ*_max_ and *σ*_min_ represent the maximum fatigue stress and the minimum fatigue stress of the CFRP sheet, respectively, *P*_k_ is the debonding load of the CFRP sheet, and σ_k_ is the debonding stress of the CFRP sheet. The crack development rate, stress ratio, and stress level of each specimen are shown in the Table 4 below.

It can be seen from Table 4 that the stress ratio and stress level (*S*) increase with the increment of the upper bound value of the fatigue loading when the lower bound value of the fatigue loading remains the same. Moreover, the stress ratio (*R*) and stress level (*S*) decrease with the increment of the lower bound value of the fatigue loading when the upper bound value of the fatigue loading stays constant. Additionally, the crack development rate (*v*_cr_) increases with the increment of the stress ratio or stress level (and decreases with the decrement of the stress ratio or stress level). Additionally, although the stress ratio (*R*) is 3.5 both for the specimen “F200-40-0.35-0.1” and “F200-40-0.7-0.2”, the stress level (*S*) and the crack development rate (*v*_cr_) are significantly different. Therefore, the stress ratio (*R*) cannot be used as a parameter to describe the crack development rate of the specimen. In this paper, the calculation model of the crack development rate with reference to the form of the Paris Law [28] has been put forward. The calculation model takes the stress level (*S*) as a parameter, as shown in Equation (6):

(6) $$\frac{da}{dN}=k\;\left(S\right){\;}^{m}$$

where *k* and *m* are undetermined coefficients affected by material properties and environmental factors. In this paper, *k* and *m* are constant because the material properties and environmental factors of all the specimens are consistent and only the stress level of fatigue load is considered. According to calculation, *k* is equal to 1.04 × 10^−2^ and *m* is equal to 4.78.

Figure 7 shows the result of the comparison between the test results and the calculated results according to Equation (6). It can be seen from Figure 7 that the test results can agree well with the calculated results, which indicates that this calculation model can be accepted to describe the relationship between crack development rate and stress level. The number of fatigue cycles during the process in which the crack length of the interface develops from *a*_0_ to *a*_c_ can be calculated by Equation (7) (deduced from Equation (6)):

(7) $$N=\int_{a_{0}}^{a_{c}}\frac{1}{k{\left(S\right)}^{m}}da$$

## 5. Analysis of Fatigue Life

### 5.1. Fatigue Life

In fatigue testing, the fatigue damage of the specimens increase with increasing number of cycles until fatigue failure occurs. The number of cycles when the fatigue failure occurs can be defined as fatigue life under the current experimental condition. Fatigue life is always expressed by *N*. It is usually be considered that fatigue failure will not occur under the current stress level if fatigue failure does not occur after two million cycles of fatigue load and the current stress level is called as the fatigue limit of the specimen. The stress level and fatigue life of each specimen are shown in the Table 5.

It can be seen from Table 5 that the fatigue life has a close relationship with the upper bound value and the lower bound value of the fatigue loading and the fatigue life decreases with the increment of stress level. A comparison of specimens F200-40-0.35-0.1, F200-40-0.4-0.1, F200-40-0.5-0.1, F200-40-0.6-0.1, F200-40-0.7-0.1, and F200-40-0.8-0.1 indicates that the fatigue lives decrease with an increase in the upper bound value of the fatigue loading when the lower bound value of the fatigue loading stays constant. Similarly, it can be seen by comparing specimens F200-40-0.7-0.1, F200-40-0.7-0.2, and F200-40-0.7-0.3 that the fatigue lives increase with an increase in the lower bound value of the fatigue loading when the upper bound value of the fatigue loading is constant.

### 5.2. S-N Curve

The *S-N* curve, first proposed by the “Father of Fatigue Tests”, A. Wohler, is the basis of fatigue life prediction and anti-fatigue design of components. The *S-N* curve represents the relationship curve between applied stress level (*S*) and fatigue life (*N*). In civil engineering research, power function form (double logarithm formula) and exponential function form (single logarithm formula) are two mature empirical expressions of the *S-N* curve [29]. It can be seen from Table 5 that the relationship between stress level (*S*) and fatigue life (*N*) is also nonlinear. In this paper, the single logarithm formula form shown in Equation (8) was used to describe the *S-N* curve of the interface between the CFRP sheets and steel plates:

(8) S=a−blgN

where *a* and *b* are undetermined coefficients. Obviously, the specimen is under a monotonic loading state when the *σ*_max_ is equal to *σ*_k_ and *σ*_min_ is equal to zero. Therefore, *N* is equal to 1 and *S* is equal to 2 as calculated by Equation (3). It can be obtained from Equation (8) that *a* is a constant and equals to 2. The effects of the material properties and the environmental factors (such as maintenance temperature) on the fatigue life of the specimen are reflected in the slope of Equation (8) *b*. In this paper, *b* is also a constant because the material properties and environmental factors of all the specimens are constant. 

The relationship curve between stress level (*S*) and fatigue life (*N*) is shown in Figure 8 through the comparative analysis of the test results in Table 5. It can be seen from Figure 8 that the fatigue life (*N*) decreases with the increment of stress level (S). The empirical formula of the *S-N* curve can be obtained through a linearity fitting, as shown in Equation (9):

(9) S= 2 - 0.263 lgN

A comparison of the test results and calculated results according to Equation (9) indicates that the test results can agree well with the calculated results, with a correlation coefficient of 0.9912. Based on the above analysis, it can be obtained that the fatigue limit under the experimental conditions in this paper is equal to 0.343 through substituting the number of cycles (*N =* 2 × 10^6^) into the Equation (9). 

Recent research [30] suggests that the Goodman-Smith Diagram can be used to perform fatigue design of FRP-strengthened structures. In this paper, Goodman-Smith Diagram is used to describe the relationship between stress level (*S*) and fatigue life (*N*). Test results are plotted in the Goodman-Smith diagram, as shown in Figure 9.

In Figure 9, the upper demarcation line is the straight line obtained by substituting the number of cycles (*N =* 2 × 10^6^) into the Equation (9). The lower demarcation line is the straight line passing through the coordinate origin and point (1,1). It can be seen from the Goodman–Smith diagram that the fatigue lives of the specimens in the region between the upper and lower demarcation lines are more than 2 million cycles and the fatigue lives of the specimens in the region above the upper demarcation line are less than 2 million cycles. The points on the upper demarcation line are the specimens whose fatigue lives are equal to 2 million cycles.

## 6. Conclusions

In this paper, experimental and theoretical research was conducted in order to investigate the bond behavior of the interface between CFRP sheets and steel plates. Two variables, namely, the upper bound value and the lower bound value of the fatigue loading, were considered in this experimental research through using double-shear specimens subjected to cyclic loading. The following conclusions can be drawn according to the research in this paper:

(1) The fatigue crack of CFRP-to-steel bonded interface propagates from the mid-span to the loaded end with the increasing numbers of cycles in the testing part. The crack development process can be divided into two stages: the first stage is a period of stable crack development and the second stage is a debonding failure period. Moreover, when the upper bound value reaches nearly 0.7*P*_k_, the impact of the stress concentration on initial crack development becomes larger.
(2) The crack development rate (*v*_cr_) increases with the increment of the stress ratio or stress level (and decreases with the decrement of the stress ratio or stress level). A calculation model of the crack development rate has been put forward and shown as Equation (6), which takes the stress level (*S*) as a parameter. The good agreement between the test results and the calculated results according to Equation (6) indicates that the model proposed in this paper can be accepted to describe the relationship between crack development rate and stress level.
(3) By comparing with the test results, it can be obtained that the fatigue life has a close relationship with the upper bound value and the lower bound value of the fatigue loading and that the fatigue life decreases with the increment of stress level.
(4) As shown in Figure 8, a comparison of the test results and calculated results according to Equation (9) indicates that the test results can agree well with the calculated results. Meanwhile, the fatigue limit calculated by Equation (9) under the experimental conditions in this paper is equal to 0.343.

## Figures and Tables

**Figure 1:** The geometry and the dimensions of the specimens. (**a**) Profile view; (**b**) top view.

**Figure 2:** Test loading device and strain acquisition system. (**a**) Test loading device; (**b**) strain acquisition system.

**Figure 3:** Typical failure modes of specimens: (**a**) specimen S200-40(1); (**b**) specimen F200-40-0.6-0.1.

**Figure 4:** The initial fatigue crack occurred at the mid-span in the testing part.

**Figure 5:** The typical strain distribution of CFRP sheets along bonding length (specimen F200-40-0.4-0.1).

**Figure 6:** The curve of interfacial crack length and number of fatigue cycles.

**Figure 7:** The comparison between the test results and the calculated results according to Equation (6).

**Figure 8:** The relationship curve between stress level (*S*) and fatigue life (*N*).

**Figure 9:** Goodman–Smith diagram for the test results obtained in the present study.

**Table 1:** Summary of material properties.

Index of Material Properties	CFRP Sheet	Adhesive	Steel Plate
Yield strength/MPa	-	-	263
Mean Tensile strength/MPa	3529.1	41.3	-
Young’s modulus /MPa	2.4 × 10^5^	2737.3	2.01 × 10^5^
Elongation/%	1.7	1.7	-
Bending strength/MPa	-	66.3	-
Shear strength (steel to steel )/MPa	-	17.7	-

**Table 2:** Details of specimens and test results.

Group	Specimen	Test Method	*b*_c_ (mm)	*l*_c_ (mm)	*P*_max_ (kN)	*P*_min_ (kN)	*R*_max_	*R*_min_	*N* (Cycles)
A	S200-40(1)	Static	40	200	27.6	-	-	-	-
	S200-40(2)	static	40	200	28.0	-	-	-	-
	F200-40-0.35-0.1	cyclic	40	200	9.73	2.78	0.35	0.1	2,982,010
	F200-40-0.4-0.1	cyclic	40	200	11.12	2.78	0.4	0.1	1,347,420
	F200-40-0.5-0.1	cyclic	40	200	13.9	2.78	0.5	0.1	187,200
	F200-40-0.6-0.1	cyclic	40	200	16.68	2.78	0.6	0.1	33,600
	F200-40-0.7-0.1	cyclic	40	200	19.46	2.78	0.7	0.1	14,020
	F200-40-0.8-0.1	cyclic	40	200	22.24	2.78	0.8	0.1	4500
B	F200-40-0.7-0.1	cyclic	40	200	19.46	2.78	0.7	0.1	14,020
	F200-40-0.7-0.2	cyclic	40	200	19.46	5.56	0.7	0.2	19,800
	F200-40-0.7-0.3	cyclic	40	200	19.46	8.34	0.7	0.3	22,400

**Table 3:** Crack development rate (*v*_cr_) of each specimen in the first stage.

Specimen	*v*_cr_ (mm/cycle)	*P*_max_/*P*_k_	*P*_min_/*P*_k_
F200-40-0.35-0.1	5.18 × 10^−5^	0.35	0.1
F200-40-0.4-0.1	9.95 × 10^−5^	0.4	0.1
F200-40-0.5-0.1	72.20 × 10^−5^	0.5	0.1
F200-40-0.6-0.1	413.22 × 10^−5^	0.6	0.1
F200-40-0.7-0.1	833.33 × 10^−5^	0.7	0.1
F200-40-0.7-0.2	549.45 × 10^−5^	0.7	0.2
F200-40-0.7-0.3	452.49 × 10^−5^	0.7	0.3

**Table 4:** Crack development rate, stress ratio and stress level of each specimen.

Specimen	*v*_cr_ (mm/cycle)	*R*	*S*
F200-40-0.35-0.1	5.18 × 10^−5^	3.5	0.32
F200-40-0.4-0.1	9.95 × 10^−5^	4.0	0.40
F200-40-0.5-0.1	72.20 × 10^−5^	5.0	0.57
F200-40-0.6-0.1	413.22 × 10^−5^	6.0	0.77
F200-40-0.7-0.1	833.33 × 10^−5^	7.0	1
F200-40-0.7-0.2	549.45 × 10^−5^	3.5	0.91
F200-40-0.7-0.3	452.49 × 10^−5^	2.3	0.80

**Table 5:** Stress level and fatigue life of each specimen.

Specimen	Stress Level *S*	Fatigue Life *N*
F200-40-0.35-0.1	0.32	2982010
F200-40-0.4-0.1	0.40	1347420
F200-40-0.5-0.1	0.57	187200
F200-40-0.6-0.1	0.77	33600
F200-40-0.7-0.1	1	14020
F200-40-0.8-0.1	1.27	4500
F200-40-0.7-0.2	0.91	19800
F200-40-0.7-0.3	0.80	22400
